The article "Ecotoxicological Assessment of Heavy Metal and Its Biochemical Effect in Fishes" was retracted in 2024. Reasons: signs of a paper mill; suspected computer-generated content; unreliable results or conclusions; concerns about the data.

# Ecotoxicological Assessment of Heavy Metal and Its Biochemical Effect in Fishes

**DOI:** 10.1155/2022/3787838

**Published:** 2022-11-26

**Authors:** Abdul Haseeb, Fozia, Ijaz Ahmad, Hidayat Ullah, Anwar Iqbal, Riaz Ullah, Bushra Abdulkarim Moharram, Alicja Kowalczyk

**Affiliations:** ^1^Department of Zoology, Kohat University of Science & Technology, Kohat 26000, Pakistan; ^2^Biochemistry Department, Khyber Medical University Institute of Medical Sciences, Kohat 26000, Pakistan; ^3^Department of Chemistry, Kohat University of Science & Technology, Kohat 26000, Pakistan; ^4^Institute of Chemical Sciences, Gomal University, Dera Ismail Khan, Pakistan; ^5^Department of Chemical Sciences, University of Lakki Marwat, Lakki Marwat, Pakistan; ^6^Department of Pharmacognosy, College of Pharmacy, King Saud University, Riyadh, Saudi Arabia; ^7^Department of Pharmacognosy, Faculty of Pharmacy, Dhaka University, Sanaa, Bangladesh; ^8^Department of Environmental Hygiene and Animal Welfare, Wrocław University of Environmental and Life Sciences, Chełmońskiego 38C, 51-630 Wrocław, Poland

## Abstract

Level of toxic heavy metal concentration like lead (Pb), chromium (Cr), cadmium (Cd), iron (Fe), copper (Cu), zinc (Zn), and nickel (Ni) in thirty-six soft and hard organs and their impact on lipid profile of *Hypophthalmichthys molitrix* and *Catla catla* fish species inhibiting in Tanda Dam reservoir were investigated. The heavy metal concentrations in water, sediment, and fish of the different regions in the reservoir were determined with atomic absorption spectrophotometer. Lipid profile was carried out by AOAC official methods. The results showed that Pb was dominant among all the heavy metals in six organs, and its maximum concentration of Pb (22.5 mg kg^−1^ and 32.9 mg kg^−1^) was observed in scales in *Hypophthalmichthys molitrix* and tail of *Catla catla*, respectively. The maximum concentrations of Cd were observed in the head, scales, fins, and gills of *Catla catla*. The bioaccumulation of heavy metals was significantly different at (*p* ≤ 0.01) within the organs and between the fish species. The lipid concentration was minimum in those organs where the concentrations of heavy metals were maximum. It is clear from the findings that heavy metal accumulation reduces the lipid content of fish. It is inevitable to monitor the Tanda Dam reservoir to safeguard human health.

## 1. Introduction

Heavy metal toxicity on fish is multidirectional and causes physiological and chemical changes in their body. The bioaccumulation of heavy metals can cause functional disturbance of organs. Accumulation of metals in various organs of fish may cause structural lesions and functional disturbances in them. A survey of heavy metal toxicity shows that the presence of heavy metals causes alterations in condition indices (condition factor and hepatosomatic index), biochemical disorders including oxidative stress and associated genotoxicity, and histopathology on aquatic organisms. At over 22,000 species, fish exhibited the supreme diversity of vertebrates. Although the fisheries sector in Pakistan is a subsector of agriculture and contributes 1% to the country's GDP. Pakistan is rich in fisheries in the marine and freshwater regions. In 2020, Pakistan's overall fish production was estimated at 701,726 metric tons, 474,025 metric tons of which were derived from marine fisheries and the remainder from inland freshwaters (Pakistan economic survey, 2019-20) [1]. The demands of the growing population eventually lead to an increase in food, so the fish industry can serve as a good source of healthy food, especially protein and lipids [2]. In human nutrition, the significance of fish is primarily due to its lipids. Fish lipids are an excellent source of polyunsaturated omega-3 fatty acids (n-3PUFA), docosahexaenoic acid (DHA), and eicosatetraenoic acid (EPA). Omega-3 polyunsaturated fatty acids are important due to their involvement in several biological processes and nutritional significance. They are important for a reduction in the cholesterol levels, decreasing the risk of heart diseases and stroke incidence, and thus, the presence of n-3 PUFAs is an essential requirement in our diet [3]. Based on this evidence, the fish are regarded as an alternative cure for heart patients [4]. In recent years, the poor wastewater treatment and practices are resulting in the contamination of water resources with heavy metals, pesticides, and inorganic fertilizers in the agricultural sector, atmospheric deposition, and geomorphological weathering of the earth's crust [5, 6], and depleting aquatic and ecosystem. As part of our diet, it is not surprising that contaminated fish can be a very dangerous source of some toxic heavy metals in the diet [7, 8]. Heavy metals have acquired the soft and hard tissues of the fish via the process of bioaccumulation. The accumulation of heavy metals in fish is used as a bioindicators to detect the concentration of heavy metals in aquatic bodies. These metals are transported from fish to their predators in the food chain [9, 10].

The article "Ecotoxicological Assessment of Heavy Metal and Its Biochemical Effect in Fishes" was retracted in 2024. Reasons: signs of a paper mill; suspected computer-generated content; unreliable results or conclusions; concerns about the data.

Heavy metal accumulation causes infertility in fish populations. Their high concentration affects the physiology and biochemical parameters of fish tissues, and heavy metals disturb body biochemistry in normal metabolic processes. These heavy metals not only accumulated in fish but also in plants in the environment and cause damage to animal and plant tissues [11–14]. In aquatic animals, heavy metals cause sublethal pathology of the liver, kidneys, reproductive, respiratory, and nervous systems [15]. Furthermore, the conversions of unsaturated fatty acids into small fragments of hydrocarbon are important for membrane lipid peroxidation. This process of peroxidation results in lipid-free radical formation, extremely toxic for carbohydrates, proteins, and lipids via the process of oxidative damage. These free radicals are regarded as reactive oxygen species and play a vital role in the inhibition of antioxidant defense mechanisms. Among the most common heavy ions in wastewater are Cd (II) and Pb (II) and responsible for grave health issues and environmental problems. Cd (II) and Pb (II) ions have a sole history of an intensive bad impact on human beings and animal health [16]. For example, Cd (II) is regarded as class I human carcinogens and Pb (II) for children compared to adults due to its higher intake by ingestion [17–20]. For example, Cd (II) is regarded as class I human carcinogens and Pb (II) for children compared to adults due to its higher intake by ingestion [21]. Several environmental issues are associated with heavy metal contamination of water [20]. Literature shows the bioaccumulation of different metals in the fishes and their resultant effects on humans. Very recently, the toxic effects of heavy metals were monitored in different families and genera of fish. It was found that the consumption of heavy metals resulted in renal impairment (Pb, Cd, and Hg), decreased cognitive function (Pb and Hg), reproductive disorder (Cd and Pb), neurological abnormalities (Hg and Pb), teratogenic disorders (Hg), and cancer (Cd) [14]. Flow sheet diagram of heavy metals in aquatic system is provided as Figure 1.

The present study explores the heavy metal concentration in two fish species *Hypophthalmichthys molitrix* and *Catla catla* and their accumulation in lipid contents in the water reservoir of Tanda Dam, a small water reservoir located in the district of Kohat, Pakistan. The reservoir is surrounded by semiarid hills of Landi Kotal and connected with river Toi in District Kohat, Khyber Pakhtunkhwa Province, Pakistan. The Tanda Dam is often used for irrigation, fishing, and picnic purposes. On July 23, 1970, it was designated as a Ramsar site for winter passage migrants stop off here as an important wetland. Local specialists in wildlife also seek to encourage cranes to use this site during migration. The area is closed off, to the captive, rare, and bred extinct animals within the province by the Khyber Pakhtunkhwa Wildlife Department. During the breeding season, the Tanda fish hatchery was established near the Tanda Dam to hatch different cyprinid species. There is rich fish fauna in the Tanda Dam, so it is a good fishing place for hunting.

The article "Ecotoxicological Assessment of Heavy Metal and Its Biochemical Effect in Fishes" was retracted in 2024. Reasons: signs of a paper mill; suspected computer-generated content; unreliable results or conclusions; concerns about the data.

## 2. Materials and Methods

### 2.1. Sample Collections

The samples of *Hypophthalmichthys molitrix* and *Catla catla* fish species, water, and sediments were collected from the Tanda Dam, Kohat, Pakistan. The water and sediment samples were collected in clear sterilized plastic bottles separately, from the inlet, outlet, and middle sides of the dam. All sediments were dried in an oven at 100°C for 24 hours. The fish specimens collected were preserved in separate bottles in a 5-percent formalin solution. To prevent deterioration, the samples were covered with sterilized polythene bags and kept at -20°C in a deep freezer until further examination. Using corrosion-resistant stainless knives, fish specimens were cut into separate sections (head, tail, abdomen, scales, fins, and gills). Each sample was placed in a separate china dish and transferred to the oven to dry at 100°C for 24 hours.

### 2.2. Preparation of Samples

The dried samples were crushed into small pieces. About 2.0 g of each sample was treated with 10 mL (concentrated HNO_3_) and 2 mL (H_2_O_2_). The samples were digested by using a hot plate (Janeway, Model-1000), and 6.0 g of each sample was subjected to a protocol of total lipids extraction as per the standard method [22].

### 2.3. Acid Digestion of Fish and Sediment Samples

Each 2.0 g dry and crushed sample of fish was weighed and transferred to a 50 mL conical flask separately, and 10 mL concentrated HNO_3_ (70%) and 2 mL H_2_O_2_ were added. The flask was heated gradually from 50 to 120°C for 30 minutes using a hot plate, and the process was continued for 12°C with the repeated addition of HNO_3_ and H_2_O_2_. The process of digestion was stopped upon the appearance of a colorless solution. The solution was placed in an open container for cooling after the complete digestion of the samples. The sample was then filtered in 50 mL clean plastic bottles with sealing plugs by Whatman Filter Paper 42. The volume of the solution was increased to 7 mL by adding 2 mL of concentrated HNO_3_. The solution was then diluted by adding 25 mL of distilled water. The samples were labeled and used for heavy metal analysis. The whole procedure was repeated until all the samples were digested and prepared for the atomic absorption spectrophotometer (Model-Analyst 400) analysis. The standard calibration for each metal element was prepared from the stock solution and analyzed at regular time intervals, to check the flow of the instrument [3]. The same procedure was adopted for sediments unless otherwise mentioned.

The article "Ecotoxicological Assessment of Heavy Metal and Its Biochemical Effect in Fishes" was retracted in 2024. Reasons: signs of a paper mill; suspected computer-generated content; unreliable results or conclusions; concerns about the data.

### 2.4. Procedure of Lipid Extraction

A 6.0 g dried and ground sample of each organ of fish were treated with 200 mL of acetone added to the sample, separately. In the continuous extractor, lipid extraction with acetone was carried out for up to 12 hours. Using a rotary evaporator, the acetone was distilled until 10-15 mL of acetone remained in the flask and was then transferred into the beaker. Finally, to make it free of oils, the flask was washed with fresh acetone. The beaker was heated to evaporate water and lipid acetone at constant temperature in a water bath. The beaker was transferred to the oven at 80°C for 1 h for complete evaporation and then shifted to cool and weighted desiccators. The sum of the extracted lipids is equal to the total lipid weight as mentioned in the following (Association of Official Analytical Collaboration (AOAC), official method of analysis, 948) [23, 24]:

(1) $$\begin{array}{c} \text{Formula lipid percentage}=\left(\frac{W_{3}-W_{1}}{W_{2}}\right)\times 100, \end{array}$$

where *W*_1_, *W*_2_, and *W*_3_ are the weight of empty beaker, sample, and lipid, respectively.

## 3. Results and Discussion

This study was performed to test the concentration of heavy metals in different parts of *Hypophthalmichthys molitrix* and *Catla catla*.  Table 1 presents the heavy metal Fe, Cu, Zn, Ni, Cd, Cr, and Pb concentrations in six body parts of *Hypophthalmichthys molitrix* and *Catla catla*. The metal Pb was found to be the highest (22.50 mg/kg) of all heavy metals in the scales of *Hypophthalmichthys molitrix*. The concentrations of all the metals in the head, gills, abdomen, tail, fins, and scales of the *Hypophthalmichthys molitrix* were as follows: the concentration of Pb was found to be maximum (15.60, 17.15, 20.20, 14.32, 20.10, and 22.50 mg/kg, respectively), while Cd showed the minimum concentration (0.032, 0.112, 0.112, 0.096, 0.064, and 0.016 mg/kg, respectively).

In the body parts of *Catla catla*, the highest heavy metal concentration was found for Pb (32.9 mg/kg) accumulated in the tail of fish, while the concentration of multiheavy metals in six body parts of *Catla catla* is found in the head, gills, abdomen, tails, fins, and scales. The concentration of Pb were found maximum (21.2, 30.0, 22.24, 32.2, 25.6, and 30.8 mg/kg, respectively), while Cd showed the minimum concentration (0.176, 0.144, 0.016, 0.08, 0.096, and 0.144 mg/kg, respectively).

Table 2 shows the concentration of heavy metals (Fe, Ni, Cu, Zn, Cd, Cr, and Pb) in water samples collected in the inlet, medium, and outlet regions of Tanda Dam water. The concentration of Pb had the maximum concentration among all heavy metals in the outlet water sample (19.802 mg/L). The reported values of Pb in the inlet, middle, and outlet regions were15.40, 18.10, and 19.802 mg/L, respectively, while Cd showed the lowest concentration among all metals, and their concentrations in the inlet, middle, and output regions were 0.144, 0.16, and 0.128 mg/L, respectively.

The article "Ecotoxicological Assessment of Heavy Metal and Its Biochemical Effect in Fishes" was retracted in 2024. Reasons: signs of a paper mill; suspected computer-generated content; unreliable results or conclusions; concerns about the data.

Table 3 represents the concentration of heavy metals in the sediment sample of the Tanda Dam. Out of all the metals present, Pb showed the highest concentration (12.5 mg/kg), while Cd has the lowest concentration (0.16 mg/kg).

Table 4 shows the comparison of heavy metals (Fe, Ni, Cu, Zn, Cd, Cr, and Pb) concentration for both species. The abdomen of *Catla catla* represented the highest concentration of Fe among all the organs of both species. The concentration of iron (Fe) in the head, tail, fins, and gills of *Hypophthalmichthys molitrix* was higher than that of the *Catla catla*, while the iron concentration in the scales and abdomen of *Catla catla* was higher than that in the *Hypophthalmichthys molitrix*. For nickel (Ni), the scales of *Catla catla* revealed the maximum concentration. Compared to the *Hypophthalmichthys molitrix*, *Catla catla* had higher concentrations of nickel in the tail, gills, fins, and scales. Only the head of the *Hypophthalmichthys molitrix* had an increased concentration of nickel than that of *Catla catla*. Copper (Cu) concentrations were higher in the scales, head, abdomen, and gills of *Catla catla* than in the *Hypophthalmichthys molitrix*. However, in the fins and tail of the *Hypophthalmichthys molitrix*, the concentration of copper was much higher than that of the *Catla catla*. The concentration of zinc in the head, tail, and abdomen of *Hypophthalmichthys molitrix* is higher than that of *Catla catla*. However, the scales, gills, and fins of the *Catla catla* have shown a greater amount of zinc than the *Hypophthalmichthys molitrix*.

In the comparison of cadmium concentration, the head, scales, gills, and fins of *Catla catla* showed higher concentration than *Hypophthalmichthys molitrix*, while the tail and abdomen of *Hypophthalmichthys molitrix* contain more cadmium concentration than *Catla catla*. The concentration of chromium in the abdomen, head, and gills of *Catla catla* was higher than that of *Hypophthalmichthys molitrix*, while the concentration of chromium in the fins and tail of *Catla catla* was lower than that of *Hypophthalmichthys molitrix*, whereas both species have an equal concentration of chromium in the scales. Lead concentration was higher in all six organs of the *Hypophthalmichthys molitrix* as compared to *Catla catla.* In *Catla catla*, the overall concentration of heavy metals, and specifically that of lead, was higher than in *Hypophthalmichthys molitrix*.

The article "Ecotoxicological Assessment of Heavy Metal and Its Biochemical Effect in Fishes" was retracted in 2024. Reasons: signs of a paper mill; suspected computer-generated content; unreliable results or conclusions; concerns about the data.

Table 5 showed the comparison of lipid percentages in both species. The highest lipid percentage (38.42 percent) was found in the head of *Hypophthalmichthys molitrix*, while scales of *Catla catla* showed the minimum lipid percentage (1.58 percent). In all six body parts, the recorded percentage of lipids was as follows: head>gills>abdomen>tail>fins>scales in both species. The overall comparison showed that the total percentage of lipids in all six organs was greater in *Hypophthalmichthys molitrix* as compared to *Catla catla*.

## 4. Discussion

The present study was conducted on two fish species of Tanda Dam Kohat, i.e., *Hypophthalmichthys molitrix* and *Catla catla*. The literature shows that the overconsumption of fish is sometimes toxic due to the concentration of heavy metals. Therefore, it was important to evaluate the heavy metals in the fish species *H. molitrix* and *Catla catla*.

The accumulation of heavy metal sand lipid contents of these two species were screened (Tables 1–5 and Figures 1–5).  Table 1 presents the concentration of multiheavy metals (iron, nickel, copper, zinc, cadmium, and lead) in the body parts of *Hypophthalmichthys molitrix* and *Catla catla* of Tanda Dam. Lead (Pb) has the highest concentration on the scales, i.e., 22.5 mg/kg, while cadmium (Cd) has the lowest concentration (0.016 mg/kg) on the scales, of all the heavy metals in the *Hypophthalmichthys molitrix*. In the head, gills, abdomen, tails, fins, and scales of the *Hypophthalmichthys molitrix*, the concentration of Pb was found maximum (15.60, 17.15, 20.20, 14.32, 20.10, and 22.50 mg/kg, respectively), while Cd showed the minimum concentration (0.032, 0.112, 0.112, 0.096, 0.064, and 0.016 mg/kg, respectively). The concentrations of lead, nickel, and iron, described by the WHO were above the permissible levels, while the concentrations of chromium, copper, zinc, and cadmium were below the permissible limits [25–28].

Table 1 also shows the heavy metal concentration in the body parts of the *Catla catla*. The highest concentration of lead (Pb) in the tail was 32.9 mg/kg, while the lowest concentration of cadmium (Cd) in the abdomen was found to be 0.016 mg/kg in all the metals present in *Catla catla*.

The recorded value of heavy metals in the head, gills, abdomen, tail, fins, and scales of *Catla catla* shows a higher concentration of lead in the head, gills, abdomen, tails, fins, and scales with values of 21.2, 30.0, 22.24, 32.2, 25.6, and 30.8 mg/kg, respectively, while Cd showed the minimum concentration (0.176, 0.144, 0.016, 0.08, 0.096, and 0.144 mg/kg, respectively) in these parts.

The article "Ecotoxicological Assessment of Heavy Metal and Its Biochemical Effect in Fishes" was retracted in 2024. Reasons: signs of a paper mill; suspected computer-generated content; unreliable results or conclusions; concerns about the data.

The concentration of lead in the body parts of *Catla catla* ranged from 32.9 to 21.2 mg/kg. The accumulation of lead, iron, and nickel was above the permissible limits, while cadmium, zinc, and chromium were below the permissible limits, and copper was within the permissible level of the WHO standard.

The present study showed that the organs of both species have different concentrations of metals.

Kalay et al. [29] reported that different species of fish have different concentrations of metals in their tissues. Also, Canli and Atli [30] reported that the concentration of heavy metals in fish varies according to their species and the aquatic environment. Kamaruzzaman et al. [31] reported a significant increase in the concentration of Pb and Cd in all heavy metals in *Cyprinus carpio* tissues.

Table 2 indicates the abundance of heavy metals in three water samples (i.e., inlet, middle, and outlet) of the Tanda Dam. Lead (Pb) has the highest concentration in the outlet water sample, i.e., 19.802 mg/kg among all metals.

The reported values for heavy metals in the inlet, middle, and outlet regions were as follows: Pb showed the highest concentration (15.40, 18.10, and 19.802 mg/L, respectively), while Cd showed the lowest concentration among all metals (0.144, 0.16, and 0.128 mg/L, respectively). In inlet water region, the order of concentration of metals was Pb>Zn>Fe>Ni>Cu>Cr>Cd, while in the middle water region, the order of concentration was Pb>Zn>Ni>Fe>Cu>Cr>Cd. In the outlet water region, the order of concentration of heavy metals was found as Pb>Ni>Zn>Fe>Cr>Cu>Cd. The concentration of all the metals in the water was above the WHO standard level, except for Cu.

Table 3 shows the concentration of iron, nickel, copper, zinc, cadmium, chromium, and lead in the sediment sample of the Tanda Dam, where lead has the highest concentration, i.e., 12.5 mg/kg, while cadmium has the lowest concentration, i.e., 0.16 mg/kg in all metals. The metal concentrations in the sediments were found in order of concentration (mg/kg) as lead> nickel>zinc>copper>iron>chromium>cadmium. The concentrations of iron, lead, cadmium, and copper were above the permissible limit, while the concentrations of zinc, chromium, and nickel were below the WHO limit. The correlation of heavy metal concentration is difficult, even between the same organs of the different species. This is due to variations of many factors, such as eating habits, whether carnivorous or herbivores, the fish habitat in deep water regions, whether surface feeder or bottom feeder, and age. Kamaruzzaman et al. [31] observed that there is a correlation between mental concentration and several basic fish variations such as fish size, age, and genetic makeup.

The article "Ecotoxicological Assessment of Heavy Metal and Its Biochemical Effect in Fishes" was retracted in 2024. Reasons: signs of a paper mill; suspected computer-generated content; unreliable results or conclusions; concerns about the data.

Table 4 shows a comparison of the concentrations of iron, nickel, copper, zinc, cadmium, chromium, and lead in the two species. The highest concentration of iron among all organs was recorded in the abdomen of *Catla catla*, i.e., 9.82 mg/kg. In the head, throat, tail, and wings, the concentration of *Hypophthalmichthys molitrix* was higher than that of *Catla catla*. The concentration of Fe in the abdomen and scales of *Catla catla* was higher than that of *Hypophthalmichthys molitrix*. Of all the organs, the highest concentration was recorded in the *Catla catla* scales, i.e., 13.74 mg/kg. Compared to the *Hypophthalmichthys molitrix*, the *Catla catla* had a higher concentration of nickel in the fins, tail, scales, and gills. Only the head of the *Hypophthalmichthys molitrix* showed a higher amount of nickel than the *Catla catla*. The concentration of copper in the head, abdomen, gills, and scales was higher in *Catla catla* as compared to *H. molitrix*, while fins and tail of *Hypophthalmichthys molitrix* showed a higher concentration of copper than *Catla catla*. Compared to the *Catla catla*, the concentration of zinc in the head, abdomen, and tail of the *Hypophthalmichthys molitrix* was higher, while the gills, scales, and fins of *Catla catla* had a higher concentration of zinc than *Hypophthalmichthys molitrix*.

Compared to *Hypophthalmichthys molitrix*, the *Catla catla* had a higher concentration of cadmium (Cd) in the head, scales, fins, and gills, while the tail and abdomen of the *Hypophthalmichthys molitrix* showed higher concentration than the *Catla catla*. In contrast to the *Hypophthalmichthys molitrix*, the *Catla catla* had a higher concentration of chromium in the head, abdomen, and gills, but the *H. molitrix* fins and tail had a higher concentration of chromium than the *Catla catla*. The scales of both species have an equal concentration of chromium. The concentration of lead was higher in all six organs of the *Catla catla* than in the *Hypophthalmichthys molitrix.* The overall concentration of heavy metals, and especially that of lead, was higher in *Catla catla* than in *Hypophthalmichthys molitrix*. This fact may be due to the reason that the Tanda Dam is filled with floods of water from the catchment area of District Orakzai and Hangu. The erosion from unexplored mountains and valleys is the cause of the higher concentration of Pb.

Table 5 represents the comparison of the complete lipid percentage in the six body parts of both species. The data shows that the lipid concentration in the head of *Hypophthalmichthys molitrix* was higher (38.42%), while the lipid concentration in the scales was the lowest (3.05%). The *Catla catla* head has the highest lipid percentage, i.e., 32.55%, while scales have the lowest percentage (1.58%). The recorded levels of lipid percentage in all six organs of *Catla catla* and *Hypophthalmichthys molitrix* were found in order of head>gills>abdomen>tail>fins>scales. According to the literature, the lipid content of fish varies over a wide range. [32–34] reported that lipids are found mainly in subcutaneous tissues of fish such as the belly flap, liver, head, muscles, and mesenteric tissues. The overall comparison showed that the total percentage of lipids in all six organs was greater in *Hypophthalmichthys molitrix* than in *Catla catla*. Although the concentration of heavy metals was higher in *Catla catla* than in *Hypophthalmichthys molitrix*, a heavy metal deposition allows biomolecules such as carbohydrates, proteins, and lipids to decline via oxidative damage. A decrease in lipid content in *Catla catla* tissues exposed to sublethal and lethal cadmium chloride concentration was reported by Sobha et al. [35]. The effect of heavy metals on lipid profiles has also been documented by Levesque et al. and Defo et al. [36, 37], Dubale and Shah [38], and Nowosad et al., Bazarsadueva et al., and Pierron et al. [39–41].

The article "Ecotoxicological Assessment of Heavy Metal and Its Biochemical Effect in Fishes" was retracted in 2024. Reasons: signs of a paper mill; suspected computer-generated content; unreliable results or conclusions; concerns about the data.

## 5. Conclusion

It was found that heavy metal accumulation decreases the lipid quantity in fish. The heavy metal content of *Catla catla* was higher than that of *Hypophthalmichthys molitrix*, although the overall percentage of lipids in *Catla catla* was smaller than that of *Hypophthalmichthys molitrix*. In both fishes, the concentration of lead, iron, and nickel was found above the permissible range as defined by the WHO, while chromium, zinc, cadmium, and copper were found below the permissible level. The concentration of these metals was found different in different body parts of both fishes as shown in Tables 1 and 2. This fact demonstrates the level of accumulation of heavy metals in different tissues among fish species. The deposition level of heavy metals also varies with the aquatic environment. Furthermore, the presence of subcutaneous tissues and their lipid content added their effect to the accumulation of heavy metals. A higher accumulation of metals and lower lipid profile was found for *Catla catla.* The presence of heavy metals is associated with oxidative stress conditions causing a lowering of the nutritional index of fish via degrading biomolecules like lipids, proteins, and carbohydrates. In water, the concentration of all metals was above the permissible range, except for copper, which was less than the permissible range. In the case of sediments, lead, iron, copper, and cadmium were determined above the permissible level, but chromium, nickel, and zinc were below the permissible range of WHO standard. Keeping in view the above findings, another detailed study is required (data unpublished) where the factors are important for the contamination of these water resources and food (fish). Moreover, the mechanistic basis of heavy metal toxicity is important to understand for essential evaluation of health hazardous assessment.

The article "Ecotoxicological Assessment of Heavy Metal and Its Biochemical Effect in Fishes" was retracted in 2024. Reasons: signs of a paper mill; suspected computer-generated content; unreliable results or conclusions; concerns about the data.

## Figures and Tables

**Figure 1:** Flow sheet diagram of heavy metals in an aquatic system.

**Figure 2:** Graphical representation of heavy metal concentration in *Hypophthalmichthys molitrix.*

**Figure 3:** Graphical representation of heavy metal concentration in water.

**Figure 4:** Comparison of heavy metal concentration (mg kg^−1^) in the body of *Hypophthalmichthys molitrix* and *Catla catla.*

**Figure 5:** Total lipids (%) in body parts of *Hypophthalmichthys molitrix* (a), *Catla catla* (b), and their comparison of total lipid (%) (c).

**Table 1:** Heavy metals concentration (mg/kg) in different body parts of *Hypophthalmichthys molitrix* and *Catla catla* collected from the Tanda Dam (mean value ± standard).

*Hypophthalmichthys molitrix*							
Heavy metals	Head	Gills	Abdomen	Tail	Fins	Scales	*p*≤
Fe	5.501 ± 0.061	6.23 ± 0.021	3.604 ± 0.103	4.126 ± 0.019	2.62 ± 0.014	2.12 ± 0.013	0.0016
Ni	3.26 ± 0.039	2.70 ± 0.013	1.648 ± 0.027	1.728 ± 0.011	3.12 ± 0.033	3.13 ± 0.011	0.0003
Cu	0.112 ± 0.014	0.864 ± 0.031	1.0721 ± 0.131	3.296 ± 0.022	3.920 ± 0.015	2.496 ± 0.005	0.0243
Zn	9.424 ± 0.82	4.016 ± 0.006	12.824 ± 0.106	10.19 ± 0.103	8.448 ± 0.018	5.968 ± 0.008	0.0012
Cd	0.032 ± 0.005	0.112 ± 0.003	0.112 ± 0.002	0.096 ± 0.001	0.064 ± 0.005	0.016 ± 0.010	0.0080
Cr	0.496 ± 0.009	0.464 ± 0.007	0.512 ± 0.002	0.544 ± 0.001	0.496 ± 0.007	0.48 ± 0.001	0.001
Pb	15.6 ± 0.051	17.15 ± 0.039	20.2 ± 0.056	14.32 ± 0.049	20.10 ± 0.127	22.5 ± 0.059	0.001
*Catla catla*							
Fe	2.912 ± 0.023	5.46 ± 0.031	9.82 ± 0.052	1.630 ± 0.002	2.52 ± 0.021	2.452 ± 0.028	0.0217
Ni	2.752 ± 0.019	4.52 ± 0.009	2.704 ± 0.02	3.808 ± 0.047	4.40 ± 0.037	13.74 ± 0.01	0.0267
Cu	2.512 ± 0.006	4.656 ± 0.096	2.96 ± 0.035	3.152 ± 0.047	2.752 ± 0.02	4.432 ± 0.112	0.0003
Zn	4.56 ± 0.002	4.848 ± 0.029	11.34 ± 0.135	10 ± 0.075	10.688 ± 0.05	9.888 ± 0.035	0.001
Cd	0.176 ± 0.004	0.144 ± 0.003	0.016 ± 0.002	0.08 ± 0.004	0.096 ± 0.004	0.144 ± 0.002	0.0056
Cr	0.528 ± 0.001	0.496 ± 0.001	0.528 ± 0.001	0.496 ± 0.002	0.352 ± 0.003	0.480 ± 0.002	0.001
Pb	21.2 ± 0.041	30.0 ± 0.094	22.24 ± 0.110	32.9 ± 0.141	25.6 ± 0.056	30.8 ± 0.095	0.001

Standard permissible limit of heavy metals in fish by WHO (FAO/WHO, 1993): Fe-0.5, Ni-0.05, Cu-3.0, Zn-30, Cd-0.5, Cr-0.6, and Pb-2.0 mg/kg.

The article "Ecotoxicological Assessment of Heavy Metal and Its Biochemical Effect in Fishes" was retracted in 2024. Reasons: signs of a paper mill; suspected computer-generated content; unreliable results or conclusions; concerns about the data.

**Table 2:** Heavy metal concentration (m min) in water samples of the Tanda Dam were collected from three different sides.

Heavy metals	Inlet	Middle	Outlet	Significant value
Fe	3.235 ± 0.058	1.942 ± 0.032	1.635 ± 0.019	*p* ≤ 0.0436
Ni	2.912 ± 0.024	3.376 ± 0.018	4.528 ± 0.012	*p* ≤ 0.0173
Cu	2.088 ± 0.109	0.928 ± 0.057	0.512 ± 0.088	*p* ≤ 0.1301
Zn	5.41 ± 0.042	4.432 ± 0.040	3.28 ± 0.035	*p* ≤ 0.0192
Cd	0.144 ± 0.004	0.16 ± 0.005	0.128 ± 0.004	*p* ≤ 0.0041
Cr	0.544 ± 0.001	0.544 ± 0.002	0.544 ± 0.001	*p* ≤ 0.001
Pb	15.40 ± 0.083	18.10 ± 0.058	19.802 ± 0.098	*p* ≤ 0.0052

The permissible limit of heavy metals in water by WHO (FAO/WHO, 1993): Fe = 0.30, Ni = 0.02, Cu = 2.00, Zn = 3.00, Cd = 0.003, Cr = 0.05, and Pb = 0.04 mg/L.

**Table 3:** Heavy metal concentration (mg/kg) in sediments collected from Tanda Dam.

Heavy metal	Sediments	Significant value
Fe	5.435 ± 0.064	*p* ≤ 0.001
Ni	8.272 ± 0.047	*p* ≤ 0.001
Cu	5.568 ± 0.266	*p* ≤ 0.0008
Zn	6.69 ± 0.078	*p* ≤ 0.001
Cd	0.16 ± 0.006	*p* ≤ 0.0005
Cr	0.528 ± 0.001	*p* ≤ 0.001
Pb	12.5 ± 0.030	*p* ≤ 0.001

Permissible limit of heavy metals in soil by WHO (FAO/WHO, 1993): Fe = 0.030, Ni = 50, Cu = 0.025, Zn = 30, Cd = 0.006, Cr = 0.8, and Pb = 0.040 mg/kg.

**Table 4:** Comparison of Fe, Ni, Cu, Zn, Cd, Cr, and Pb concentrations (mg/kg) in the body of *Hypophthalmichthys molitrix* and *Catla catla* collected from the water of the Tanda Dam (mean value ± standard).

Heavy metals	Parameters	*H. molitrix*	*Catla catla*	*p*≤
		Temperature 273 K		
Fe	Head	5.50 ± 0.06	2.91 ± 0.02	0.1901
	Gills	6.2 ± 0.02	5.46 ± 0.03	0.0419
	Abdomen	3.60 ± 0.10	9.82 ± 0.05	0.2761
	Tail	4.13 ± 0.02	1.63 ± 0.01	0.2605
	Fins	2.62 ± 0.014	2.52 ± 0.02	0.0124
	Scales	2.12 ± 0.013	2.45 ± 0.03	0.0461

Ni	Head	3.26 ± 0.04	2.75 ± 0.02	0.0537
	Gills	2.70 ± 0.02	4.52 ± 0.01	0.0431
	Abdomen	1.65 ± 0.03	2.70 ± 0.02	0.1529
	Tail	1.728 ± 0.01	3.80 ± 0.05	0.2288
	Fins	3.12 ± 0.03	4.40 ± 0.04	0.1073
	Scales	3.13 ± 0.01	13.74 ± 0.01	0.3574

Cu	Head	0.11 ± 0.01	22.51 ± 0.01	0.4716
	Gills	0.86 ± 0.03	4.66 ± 0.10	0.3832
	Abdomen	1.072 ± 0.13	2.96 ± 0.04	0.2788
	Tail	3.30 ± 0.02	3.15 ± 0.05	0.0142
	Fins	3.92 ± 0.02	2.75 ± 0.02	0.1103
	Scales	2.50 ± 0.01	4.43 ± 0.11	0.1735

Zn	Head	9.42 ± 0.82	4.56 ± 0.01	0.2131
	Gills	4.02 ± 0.01	4.85 ± 0.03	0.0596
	Abdomen	12.82 ± 0.11	11.34 ± 0.14	0.0390
	Tail	10.19 ± 0.10	10.00 ± 0.08	0.0060
	Fins	8.45 ± 0.018	10.69 ± 0.05	0.0742
	Scales	5.97 ± 0.01	9.89 ± 0.04	0.1543

Cd	Head	0.03 ± 0.01	0.18 ± 0.01	0.3855
	Gills	0.11 ± 0.01	0.14 ± 0.03	0.0792
	Abdomen	0.11 ± 0.02	0.02 ± 0.02	0.4097
	Tail	0.10 ± 0.01	0.08 ± 0.02	0.0577
	Fins	0.06 ± 0.05	0.10 ± 0.04	0.1257
	Scales	0.02 ± 0.01	0.14 ± 0.02	0.4296

Cr	Head	0.50 ± 0.01	0.53 ± 0.01	0.0199
	Gills	0.46 ± 0.01	0.50 ± 0.01	0.0212
	Abdomen	0.51 ± 0.02	0.53 ± 0.01	0.0098
	Tail	0.54 ± 0.02	0.50 ± 0.02	0.0294
	Fins	0.50 ± 0.01	0.35 ± 0.03	0.1071
	Scales	0.48 ± 0.01	0.48 ± 0.02	0

Pb	Head	15.60 ± 0.05	21.20 ± 0.04	0.0961
	Gills	17.15 ± 0.04	30.00 ± 0.09	0.1694
	Abdomen	20.20 ± 0.06	22.24 ± 0.11	0.0306
	Tail	14.32 ± 0.05	32.90 ± 0.14	0.2387
	Fins	20.10 ± 0.13	25.60 ± 0.06	0.0763
	Scales	22.50 ± 0.06	30.80 ± 0.10	0.0983

The article "Ecotoxicological Assessment of Heavy Metal and Its Biochemical Effect in Fishes" was retracted in 2024. Reasons: signs of a paper mill; suspected computer-generated content; unreliable results or conclusions; concerns about the data.

**Table 5:** Total lipids % and age in different body parts of *Hypophthalmichthys molitrix*, *Catla catla,* and their comparison collected from the water of Tanda Dam.

Organs	Fish species		Comparison		
	*Hypophthalmichthys molitrix* lipids (%)	*Catla catla* lipids (%)	Lipid % of *H. molitrix*	Lipid % of *Catla catla*	*p*≤
Head	38.42	32.55	38.42	32.55	0.0525
Gills	23.47	22.08	23.47	22.08	0.0194
Abdomen	19.73	16.00	19.73	16.00	0.0662
Tail	16.51	14.73	16.51	14.73	0.0362
Fins	11.75	6.37	11.75	6.37	0.1837
Scales	3.05	1.58	3.05	1.58	0.1957
*p* value	0.0118	0.0184	—	—	—

## Data Availability

All available data are incorporated in the MS.
